# The Role of BRAF Inhibitors in the Management of Ameloblastoma: A Literature Review

**DOI:** 10.7759/cureus.47682

**Published:** 2023-10-25

**Authors:** Arindam Malakar, V. Raj Kumar, Priya Yadav, Vishal Bhardwaj, Chuimee Gogoi Barua, Gourika Bhardwaj

**Affiliations:** 1 Oral and Maxillofacial Surgery, Prabhu Dayal Memorial (PDM) Dental College and Research Institute, PDM University, Bahadurgarh, IND; 2 Periodontics, Employees’ State Insurance Corporation (ESIC) Dental College and Hospital, Delhi, IND; 3 Oral and Maxillofacial Surgery, Career Postgraduate Institute of Dental Sciences and Hospital, Lucknow, IND; 4 Dentistry, Prabhu Dayal Memorial (PDM) Dental College and Research Institute, PDM University, Bahadurgarh, IND

**Keywords:** mapk pathway, targeted therapy, braf v600e mutations, ameloblastoma, braf mutation

## Abstract

Ameloblastoma is one of the most prevalent but enigmatic benign odontogenic tumors of the jaw, accounting for approximately 10% of all maxillary and mandibular tumors. This neoplasia is distinguished by exhibiting several clinical and histological variants along with several mutations that affect its behavior. The ameloblastoma treatment plan is determined by the tumor's size, anatomical location, histologic variant, and anatomical involvement. On chromosome 7, there is a proto-oncogene called BRAF. When BRAF is mutated, it becomes an oncogene and continuously produces proteins like MEK and ERK, members of mitogen-activated protein kinase (MAPK). In the signaling pathway, these proteins activate transcription factor inside the nucleus that helps in cell division and growth. Numerous neoplasms have been linked to more than 40 BRAF mutations. The most common one is BRAF proto-oncogene serine/threonine kinase (BRAF) V600E, whose treatment has been linked to a positive outcome. BRAF inhibitors like vemurafenib, dabrafenib, and sorafenib have shown excellent results, especially in metastatic ameloblastoma.

BRAF, particularly in the case of metastatic ameloblastoma, inhibitors such as vemurafenib, dabrafenib, and sorafenib, has demonstrated outstanding results. Targeted therapies have been employed as adjuvant therapies to enhance cosmetic outcomes, even though no reports of serial cases demonstrate their effectiveness in ameloblastomas. In the treatment of ameloblastomas, the identification of BRAF V600E and additional mutations as the prime targeted therapies has proven to be a significant breakthrough where surgical treatment was contraindicated. In this article, we review the presence of BRAF V600E mutations, their inhibitors, and targeted therapies in ameloblastoma.

## Introduction and background

According to WHO, ameloblastoma is a benign intraosseous neoplasm originating from the odontogenic epithelium. It is characterized by its locally invasive growth pattern and tendency to recur. Comprised of odontogenic ectomesenchyme and mature fibrous stroma in the epithelium, ameloblastoma is considered an aggressive neoplasm [1]. Predominantly affecting young individuals, this tumor commonly manifests in the mandible, accounting for approximately 80% of cases. Incomplete removal often leads to recurrence, necessitating total bone excision with an adequate safety margin, known as segmental or marginal osteotomy, as the conventional treatment approach [2].

However, the conventional surgical management of massive ameloblastoma has presented significant challenges, such as cosmetic abnormalities, functional impairments, and psychological distress. The most recent WHO classification identifies four subtypes of ameloblastoma: solid/multicystic ameloblastoma, unicystic ameloblastoma, peripheral ameloblastoma, and desmoplastic ameloblastoma [3]. Surgery remains the preferred treatment modality, ranging from drastic measures like enucleation or curettage to more conservative approaches. Both options, however, entail considerable morbidity, with the former associated with high recurrence rates of up to 90% [2]. Recent advancements in understanding the molecular mechanisms underlying ameloblastoma development have revealed new therapeutic opportunities. In particular, studies conducted by Kurppa et al., Brown et al., and Sweeney et al. from 2014 onward have revealed alterations in the mitogen-activated protein kinase (MAPK) cascade, with the activating mutation BRAF V600E being identified in 40-80% of cases [4]. This mutation plays a crucial role in the pathogenesis of ameloblastoma, which can metastasize and have significant clinical implications.

The global incidence of ameloblastoma is approximately 0.5 cases per million people, with higher prevalence observed in China and Africa, where it comprises 10% of all cystic and tumor lesions in the maxilla and mandible. Surgical resection remains the primary therapeutic option and leads to the complete eradication of the neoplasm in the majority of cases. However, adjuvant therapies, including radiotherapy and chemotherapy, are employed when ameloblastoma recurs or presents as metastatic ameloblastoma or ameloblastic carcinoma. Nonetheless, employing these adjuvant therapies alone without surgical intervention has resulted in uncertain outcomes and elevated recurrence rates, leading to considerable controversy [1].

The management of ameloblastoma has witnessed significant advancements in recent years, particularly in the realm of targeted therapies aimed at specific mutations present in the tumor. One of the most prevalent mutations identified in ameloblastoma is the BRAF proto-oncogene serine/threonine kinase (BRAF) V600E mutation, and targeted treatment strategies against this mutation have shown promising outcomes [1]. Targeted therapies are designed to selectively inhibit the specific molecular alterations driving tumor growth, thereby offering a more precise and effective approach to treatment. In the case of ameloblastoma, the BRAF V600E mutation has emerged as a potential therapeutic target. Numerous studies have demonstrated that patients harboring this mutation tend to respond favorably to targeted therapies.

BRAF inhibitors specifically target the aberrant BRAF signaling pathway and have shown promising results in preclinical and early clinical studies. These medications work by blocking the activity of the mutated BRAF protein, effectively hindering its signaling cascade and impeding tumor growth. By directly addressing the underlying genetic alteration, targeted therapies hold the potential to improve treatment outcomes and minimize the adverse effects associated with conventional surgical approaches [2]. However, it is important to note that targeted therapies are still in the early stages of investigation for ameloblastoma, and more research is needed to fully understand their long-term efficacy, safety profile, and optimal usage. Clinical trials are currently underway to evaluate the effectiveness of BRAF inhibitors and other targeted agents in the management of ameloblastoma, aiming to further refine treatment strategies and optimize patient outcomes.

## Review

It was discovered in 2002 that BRAF mutations are present in certain human cancers. Mutations in BRAF can also lead to birth defects when inherited [5]. In the realm of cancer therapy, medications have been created to combat cancers that are fueled by BRAF mutations. For the treatment of late-stage melanoma, the FDA has approved two such drugs: vemurafenib and dabrafenib. Vemurafenib, in particular, was the first drug developed through fragment-based drug discovery to receive approval [6]. BRAF belongs to the Raf kinase family, which plays a role in the MAP kinase/ERK signaling pathway. This pathway influences processes such as cell division, differentiation, and secretion. The BRAF protein consists of three conserved domains characteristic of the Raf kinase family: conserved region 1 (CR1), a self-regulatory domain that binds Ras-GTP; conserved region 2 (CR2), a serine-rich hinge region; and conserved region 3 (CR3), a catalytic protein kinase domain responsible for phosphorylating protein substrates. As a serine/threonine-specific protein kinase, BRAF catalyzes the phosphorylation of serine and threonine residues on target proteins using ATP as a substrate [7]. This process results in the production of ADP and a phosphorylated protein. Activation of BRAF as an enzyme requires binding to Ras-GTP. Once activated, the catalytic core of BRAF phosphorylates protein substrates by facilitating the attack of the substrate's serine or threonine hydroxyl group on the γ-phosphate group of ATP through a bimolecular nucleophilic substitution mechanism.

More than 30 mutations of the BRAF gene have been identified in association with human cancers. The frequency of these mutations varies across different types of cancers. BRAF mutations are highly prevalent in melanomas and nevi, with more than 80% of cases exhibiting these mutations. In contrast, other tumors, such as lung cancers and colorectal cancer, show a lower frequency of BRAF mutations, ranging from 0% to 18% and 5%, respectively [8]. The most common mutation found in approximately 90% of cases involves a substitution of thymine with adenine at nucleotide 1799. This results in the substitution of valine with glutamate at codon 600, known as the V600E mutation [9]. The V600E mutation has been observed in various cancers, including papillary thyroid carcinoma, colorectal cancer, melanoma, non-small-cell lung cancer, Langerhans cell histiocytosis, and hairy cell leukemia. It is also detected in a significant proportion of ameloblastomas, a locally infiltrative odontogenic neoplasm. Additionally, the V600E mutation has been associated with certain cases of papillary craniopharyngioma development [10,11].

Other mutations have also been identified, including R461I, I462S, G463E, G463V, G465A, G465E, G465V, G468A, G468E, G469R, N580S, E585K, D593V, F594L, G595R, L596V, T598I, V599D, V599E, V599K, V599R, V600K, A727V, and more. These mutations cluster in two regions: the glycine-rich P loop of the N lobe and the activation segment and flanking regions. These mutations lead to a change in the conformation of the activation segment, transitioning it from an inactive state to an active state. The specific type of mutation can affect the kinase activity of BRAF toward MEK, with most mutants showing enhanced kinase activity. However, some mutants act through different mechanisms, reducing their activity toward MEK but activating wild-type CRAF, which subsequently signals to ERK [12]. These BRAF mutations and their impact on protein function are crucial for developing targeted therapies for cancers. By targeting the specific altered signaling pathways associated with these mutations, researchers aim to improve treatment outcomes for patients with BRAF-mutated cancers.

BRAF V600E: a genetic alteration

BRAF V600E is a specific mutation of the BRAF gene that has been extensively studied in various neoplasms, including ameloblastoma, unicystic ameloblastoma, acanthomatous ameloblastoma, plexiform ameloblastoma, and metastatic ameloblastoma. The BRAF gene plays a crucial role in cellular mechanisms, such as metabolism and proliferation. The most frequent mutation occurs at residue 600 of the BRAF gene, where valine is replaced by glutamine (V600E). This mutation leads to the constitutive activation of the MEK/ERK signaling pathway in tumors. In the case of ameloblastomas, the presence of the BRAF V600E mutation was first described by Brown et al. and Kurppa et al. These studies highlighted its influence on resistance to targeted therapies, particularly those targeting EGF receptors. Additionally, Jhamb et al. described the association between BRAF and the RAS/MAPK pathway in the pathogenesis of ameloblastoma [1].

Fujii et al. reported that the oncogenic BRAF V600E mutation led to the activation of the MAPK pathway, resulting in successful treatment with a BRAF inhibitor. Furthermore, they observed that the expression of ADP ribosylation factor (ARF)-like 4c (ARL4C) was induced by a combination of signals from the EGF-MAPK pathway and Wnt/β-catenin signaling, which in turn initiated epithelial morphogenesis. It was noted that when ARL4C was overexpressed due to alterations in the EGF/RAS-MAPK pathway and Wnt/β-catenin signaling, it promoted the development of tumorigenic characteristics. Additionally, there seemed to be potential cooperation between the RAF1-MEK/ERK-ARL4C axis and the BRAF V600E-MEK/ERK pathway, contributing to the advancement of ameloblastoma [13].

Sweeney et al. found the BRAF V600E mutation in 46% of analyzed ameloblastoma cases, along with other variants of the BRAF mutation (such as L597R) associated with increased kinase activity. Associations with other mutations, such as SMO and FGFR2, have also been reported in maxillary ameloblastomas. The detection of BRAF V600E in ameloblastoma is commonly performed using immunohistochemical techniques with specific antibodies. Its expression has been associated with recurrence, osseous disruptions, and certain radiographic patterns. The presence of the BRAF mutation is also linked to clinical behavior in ameloblastomas, often being associated with other mutations and occurring more frequently in younger patients [14].

In the research conducted by Brown et al., mutations were observed in several genes, including BRAF, KRAS, NRAS,

FGFR2, SMO, SMARCB1, CTNNB1, and PIK3CA. Notably, the BRAF V600E mutation emerged as the most frequently occurring mutation, accounting for 62% of the cases [15]. Similarly, in a study published by Diniz et al. in 2015, it was revealed that the BRAF V600E mutation was detected in 82% of the studied cases. In a more recent investigation by Girardi et al. involving 62 patients with ameloblastoma, mutations were identified in 57 of these individuals, representing 92% of the cohort. Of these mutations, the BRAF V600E mutation stood out as the most prevalent, being present in 60% of the patients. Additionally, SMO mutations were identified in 14% of the patients [4]. In the case of unicystic ameloblastoma, no additional mutations to BRAF V600E have been reported. This difference suggests that BRAF expression may occur earlier in the tumorigenesis of ameloblastomas, and additional mutations may be acquired during tumor evolution. Alternatively, unicystic ameloblastoma may be a precursor neoplasia of ameloblastoma, with mutated BRAF present from the beginning of the pathology. Acanthomatous ameloblastoma, classified as an aggressive ameloblastic tumor with a tendency to metastasize, has also been found to harbor BRAF mutations similar to ameloblastoma. However, in the analysis, a lower number of acanthomatous ameloblastoma cases were reported with the BRAF V600E mutation compared to unicystic ameloblastoma [1].

Gonzalez-Gonzalez et al. stated that in plexiform ameloblastoma cases, a high percentage of BRAF V600E mutations were reported, but the small number of cases limits the generalization of the findings [1]. Plexiform ameloblastoma, although similar to intraosseous ameloblastoma histologically, is less aggressive due to its location. Metastatic ameloblastoma, a rare ameloblastoma that develops metastases despite its benign appearance, was found to have a higher prevalence of BRAF V600E mutations compared to other ameloblastomas. This suggests that secondary mutations of BRAF V600E may be exclusive to ameloblastoma. Metastatic ameloblastoma is an uncommon tumor, and its outcomes depend on the presence of metastatic nests and surgical viability [1].

Overall, the BRAF V600E mutation has emerged as a predictive, diagnostic, and prognostic biomarker in ameloblastomas. Further studies are needed to explore the functional implications of additional BRAF mutations, their relationship with histological pathways and tumor behaviors, and their potential role in treatment resistance. The BRAF V600E mutation in ameloblastomas is more frequent in the mandible, particularly in the body, ramus, and symphysis [16]. The ratio of BRAF V600E mutations in the mandible compared to the maxilla is approximately 21:1, although some cases with the mutation do not have a specific anatomical location.

Gultekin et al. found from the studied cases that the majority (93.7%) of BRAF V600E mutations did not have additional mutations, while 6.23% of cases had multiple mutations. This suggests that treatment targeting BRAF V600E alone may be successful in many cases. Interestingly, the percentage of cases with multiple mutations was higher in the maxilla (27.7%) compared to the mandible (4.3%). This finding indicates that combined therapies may be more effective for maxillary tumors, as the most frequently observed secondary mutation in the maxilla was SMO. Isolated SMO mutations can also be present, potentially requiring a modification in the treatment strategy. Tumors with multiple mutations are associated with a higher risk of recurrence [17].

Additional mutations identified in mandibular ameloblastomas included JAK P132T, SMO, SMARCB1, PIK3CA, and CTNNB1. In maxillary ameloblastomas, additional mutations included BRAF L597R, FGFR2, PIK3CA, and SMO. Other secondary mutations without specified anatomical locations included BRAF G606E, CTNNB1, CDKN2A, and PTEN. The presence of JAK3 P132T mutation in ameloblastomas has not been previously associated with the condition. However, this gene has been studied in other neoplasms, such as head and neck squamous cell carcinoma and leukemias [18].

Table 1 shows the gene mutations of ameloblastoma by various research.

**Table 1:** Gene mutations of ameloblastoma by various research N/A: not available

Journal/references	Year	Number of ameloblastoma	Gene mutation	Gene involved	Signaling pathway
Pereira et al. [3]	2016	8	V600E	BRAF (5)	MAPK/ERK
Sweeney et al. [14]	2014	28	L412F (10)	SMO (11)	Hedgehog
Brown et al. [15]	2014	50	V600E	BRAF (31)	MAPK/ERK
Heikinheimo et al. [16]	2018	73	V600E	BRAF (58)	MAPK/ERK
Shibata et al. [19]	2002	12	C238Y	TP53 (1)	p53
Sekine et al. [20]	2003	20	S45P	CTNNB1 (1)	Wnt/β-catenin
Kumamoto et al. [21]	2004	10	No mutation	TP53 (0)	p53
Kawabata et al. [22]	2005	14	N/A	CTNNB1 (1)	Wnt/β-catenin
Oikawa et al. [23]	2013	18	No mutation	EGFR (0)	EGFR
Kurppa et al. [24]	2014	24	V600E	BRAF (15)	MAPK/ERK
Diniz et al. [25]	2015	17	V600E	BRAF (14)	MAPK/ERK
Brunner et al. [26]	2015	19	V600E	BRAF (14)	MAPK/ERK
Li et al. [27]	2016	30	N/A	APC (ND)	Wnt/β-catenin
Xia et al. [28]	2019	5	V600E	BRAF (3)	MAPK/ERK
Oh et al. [29]	2019	30	V600E	BRAF (27)	MAPK/ERK

BRAF inhibitors and mechanism of action

Vemurafenib, dabrafenib, and encorafenib, known as BRAF inhibitors, are employed in the treatment of patients afflicted with BRAF-mutant melanoma. These medications specifically target BRAF kinase, disrupting the functioning of the MAPK signaling pathway, which plays a pivotal role in regulating the growth and viability of melanoma cells. In addition to their precise molecular targeting, BRAF inhibitors exert immunomodulatory effects. Typically, the BRAF protein is activated through interaction with the G-protein RAS. Notably, mutations in RAS encompassing variants, such as KRAS, NRAS, and HRAS, have been identified in a significant portion of ameloblastoma cases, reaching up to 20%. Intriguingly, this mutation appears to be specific to ameloblastic tumors, hinting at its potential utility as a diagnostic marker [30].

Kinase Inhibition

Approved for treating advanced melanoma patients with BRAF V600 mutations, drugs like vemurafenib, dabrafenib, and encorafenib serve as oral small-molecule inhibitors that specifically target BRAF kinase. By halting BRAF activity, they disrupt the MAPK signaling pathway responsible for governing melanoma cell proliferation and survival.

Immune System Enhancement (Tumor Environment)

BRAF inhibitors possess the ability to counteract some of the immune-suppressing effects commonly associated with the BRAF-mutant tumor microenvironment. Firstly, these inhibitors promote the creation of an immune-stimulating environment within BRAF-mutant melanomas. Secondly, they facilitate greater infiltration of T cells into the tumor microenvironment. Lastly, BRAF inhibitors enhance the effectiveness of effector T cells [30]. Table 2 shows the types of BRAF inhibitors.

**Table 2:** Types of BRAF inhibitors

Type I	Type II
Vemurafenib	Sorafenib
Dabrafenib	Regorafenib
LGX 818	XL 281
PLX 4720	RAF 265
SB-590885	

In vitro studies have shown promising results for the therapeutic use of treatments targeting the BRAF V600E mutation in ameloblastomas. Vemurafenib, a BRAF inhibitor, has been evaluated in the ameloblastoma-1 cell line and demonstrated a reduction in cell proliferation and activation of the MAPK signaling pathway. This suggests that vemurafenib could be a potential alternative for the treatment of ameloblastomas, especially in cases where surgical treatment is associated with significant facial deformities and frequent recurrences. Vemurafenib is recommended as an alternative treatment for locally aggressive tumors in patients who are not candidates for surgery [15].

Exploration into combination therapies has been ongoing, including the utilization of vemurafenib (a BRAF inhibitor) alongside trametinib (a MEK inhibitor). Notably, some documented cases have displayed highly favorable outcomes with this combined approach, especially in instances of metastatic ameloblastoma. While there's a notable absence of reports indicating the outright success of targeted therapies in treating ameloblastomas, they have found application as adjuvant or neoadjuvant therapies aimed at enhancing treatment results, functional mobility, and cosmetic outcomes. However, it is worth mentioning that the utilization of targeted therapies in the context of ameloblastomas has remained relatively limited so far [15].

In the research conducted by Kaye et al., a case of ameloblastoma with a history of multiple recurrences following radical surgeries was documented. This particular case went on to develop lung metastasis. Notably, the presence of the BRAF V600E mutation was detected. To address the situation, a treatment regimen featuring dabrafenib (a BRAF inhibitor) and trametinib (a MEK inhibitor) was initiated. Remarkably, this approach resulted in the complete alleviation of symptoms and an exceptionally positive radiological response [31].

Similarly, Tan et al. reported another case involving recurrent ameloblastoma, which had resurfaced following a conservative procedure. In this instance, treatment involving the administration of dabrafenib led to a remarkable reduction in tumor size. Consequently, the patient became eligible for subsequent radical resection of the remaining lesion [32].

Lastly, Faden et al. described a case concerning an 83-year-old woman who had recurrent ameloblastoma featuring the BRAF V600E mutation. Due to existing comorbidities, further surgical intervention was deemed unsuitable for this patient. Instead, she received dabrafenib treatment, resulting in a significant reduction in the lesion size and a sustained response that endured for 12 months [33].

## Conclusions

In conclusion, BRAF inhibitor therapy represents a significant advancement in the management of ameloblastomas, offering an alternative treatment approach for patients who are not suitable candidates for surgical interventions due to the risk of significant facial deformities and recurrent recurrences. However, it is important to note that the use of BRAF inhibitor therapies in ameloblastomas is still in its early stages. Further research is required to validate the efficacy, optimize treatment protocols, minimize toxicities, and improve overall patient outcomes. Continued investigation into targeted therapies and the development of personalized treatment strategies hold great promise for improving the management and prognosis of ameloblastomas in the future.
